RETRACTED

# Anti-hyperalgesic properties of a flavanone derivative Poncirin in acute and chronic inflammatory pain models in mice

**DOI:** 10.1186/s40360-019-0335-5

**Published:** 2019-09-11

**Authors:** Ruqayya Afridi, Ashraf Ullah Khan, Sidra Khalid, Bushra Shal, Hina Rasheed, Muhammad Zia Ullah, Omer Shehzad, Yeong Shik Kim, Salman Khan

**Affiliations:** 1 Department of Pharmacy, Faculty of Biological Sciences, Quaid-i-Azam University, Islamabad, Pakistan; 2 Department of Pharmacy, Abdul Wali Khan University, Mardan, Pakistan; 3 College of Pharmacy, Seoul National University, Seoul, 151-742 South Korea

**Keywords:** Poncirin, Inflammatory pain, Cytokines, Hyperalgesia, Allodynia

## Abstract

**Background:**

Poncirin is flavanone derivative (isolated from *Poncirus trifoliata*) with known pharmacological activities such as anti-tumor, anti-osteoporotic, anti-inflammatory and anti-colitic. The present study aimed to explore the anti-allodynic and anti-hyperalgesic potentials of poncirin in murine models of inflammatory pain.

**Methods:**

The analgesic potential of poncirin was evaluated in formalin-, acetic acid-, carrageenan- and Complete Freund’s Adjuvant (CFA)-induced inflammatory pain models in mice. Anti-allodynic and anti-hyperalgesic activities were measured using Von Frey filaments, Randall Selitto, hotplate and cold acetone tests. The serum nitrite levels were determined using Griess reagent. The Quantitative Real-time PCR (qRT-PCR) was performed to assess the effect of poncirin on mRNA expression levels of inflammatory cytokines and anti-oxidant enzymes.

**Results:**

Intraperitoneal administration of poncirin (30 mg/kg) markedly reduced the pain behavior in both acetic acid-induced visceral pain and formalin-induced tonic pain models used as preliminary screening tools. The poncirin (30 mg/kg) treatment considerably inhibited the mechanical hyperalgesia and allodynia as well as thermal hyperalgesia and cold allodynia. The qRT-PCR analysis showed noticeable inhibition of pro-inflammatory cytokines (mRNA expression levels of TNF-α, IL-1β and IL-6) (*p* < 0.05) in poncirin treated group. Similarly, poncirin treatment also enhanced the mRNA expressions levels of anti-oxidant enzymes such as transcription factor such as nuclear factor (erythroid-derived 2)-like 2 (Nrf2) (*p* < 0.05), heme oxygenase (HO-1) (*p* < 0.05) and superoxide dismutase (SOD2) (*p* < 0.05). Chronic treatment of poncirin for 6 days did not confer any significant hepatic and renal toxicity. Furthermore, poncirin treatment did not altered the motor coordination and muscle strength in CFA-induced chronic inflammatory pain model.

**Conclusion:**

The present study demonstrated that poncirin treatment significantly reduced pain behaviors in all experimental models of inflammatory pain, suggesting the promising analgesic potential of poncirin in inflammatory pain conditions.

RETRACTED

**Electronic supplementary material:**

The online version of this article (10.1186/s40360-019-0335-5) contains supplementary material, which is available to authorized users.

## Background

Pain is the major protective response that is initiated by peripheral sensory neurons to protect the organism from any harm by infection or tissue injury [1]. Pain helps the body to take corrective actions in the presence of any noxious stimuli. However, the presence of pain is not always beneficial, in certain clinical scenarios; pain increases the suffering when there is a dysfunction in nociceptive pathways for example in neuropathic pain and abnormal central amplifications syndromes [1]. Inflammatory pain results whenever injury to the tissues ensues, causing the release of inflammatory mediators, which decreases pain threshold by increasing the transduction of painful stimuli [2]. These inflammatory mediators including tumor necrosis factor-α (TNF-α), interleukin-1β (IL-1β) and IL-6, reduces pain threshold by directly sensitizing nociceptors and causing its increased responsiveness leading to a state of hyperalgesia and allodynia [3, 4]. In addition to directly activating nociceptive fibers, these cytokines also potentiate the inflammatory responses and increase the release of proalgesic agents including nerve growth factor (NGF), extracellular protons, bradykinin, and prostaglandins, resulting in pain hypersensitivity [5]. These inflammatory mediators are also linked with an increased transcription of various inflammatory genes through transcription factors including mitogen activated protein kinases (MAPKs), cAMP response element-binding protein (CREB) and Nuclear factor kappa B (NF-κB), which further aggravates the immune and pain responses by altering the neuronal threshold [5–7].

Although, painful conditions either acute or chronic inflammatory pain, constitute a major health problem. There is still need for safe and effective therapeutic options. For example, non-steroidal anti-inflammatory drugs (NSAIDs) are widely used for the management of inflammatory pain conditions, are unable to completely abolish pain and are associated with several serious adverse effects including gastrointestinal bleeding and renal toxicity [8]. On the other hand, opioid analgesic represents a potent class of analgesics are also associated with major adverse effects including physical and psychological dependence, lethargy, euphoria, respiratory depression [8]. Current therapies available for treating acute and chronic inflammatory are inadequate and there is a need of newer and safer analgesics and anti-inflammatory drugs, that have better efficacy and tolerability [9, 10].

RETRACTED

Medicinal plants have been used for centuries for pain management, which can be used as a potential source for the development of novel analgesics for treating pain [11]. Poncirin is a flavanone derivative obtained from dried immature fruits of *Poncirus trifoliata*. *Poncirus trifoliata* belongs to genus Citrus, which have been used in Chinese medicine for the treatment of asthma and inflammation [12]. Several studies reported that poncirin exhibit anti-inflammatory [13], anti-tumor [14], anti-osteoporotic activity [15] and anti-colitic properties (Kang and Kim 2016). Therefore, in the present study various animal models of pain were carried out to assess the anti-allodynic, anti-hyperalgesic and anti-nociceptive properties of poncirin as a potential new analgesic to treat different types of inflammatory pain.

## Methods

### Chemicals and reagents

Carrageenan, Complete Freund’s adjuvant (CFA), formalin, acetic acid, dexamethasone, Griess reagent, acetone, piroxicam, and poncirin were obtained from Sigma chemical company (St. Louis, MO, USA). Trizol reagent was obtained from Invitrogen (USA).

### Ethics approval and consent to participate

All procedures were complied with “Animal care guidelines of QAU” Islamabad. The study was also approved by Bioethical Committee (*Approval No: BEC-FBS-QAU 2017–2*) of QAU University, Islamabad. All the experiments were designed to cause minimum harm to animals.

### Animals

All experiments were performed on male albino (BALB/c mice, 4–5 weeks of age, weighing 25–30 g), purchased from National Institute of Health (NIH), Islamabad, Pakistan. All behavioral assays were carried out in pathogen-free environment of laboratory of Pharmacology, Department of Pharmacy, QAU, Islamabad, Pakistan. Seven animals were housed per cage in controlled temperature and humidity, with free access to food and water. All experiments were performed between 8:00 a.m. to 6:00 p.m. During the current study, fresh/separate set of animals were procured for each model (acetic acid, formalin, carrageenan and CFA) and used once as per institutional ethical guidelines.

### Experimental groups and treatment protocols

The animals were randomly arranged into various groups and each group consists of 6–7 animals. The vehicle control received only normal saline with 2% DMSO and no other treatment or inducer was given. The negative control group received either acetic acid, formalin, Carrageenan or CFA and no other treatment was administered. The positive control either received Piroxicam (in case of formalin and acetic acid-induced models), while dexamethasone was administered in case of the Carrageenan and CFA-induced inflammatory models. The treatment control received the poncirin at three different doses such as 5 mg/kg, 15 mg/kg and 30 mg/kg in case of formalin, acetic acid and Carrageenan-induced models, while only 30 mg/kg dose was administered to only CFA-induced models. The inclusion and exclusion criteria was followed as reported previously [16]. The animals were anesthetized with the Xylazine + ketamine injection (16 mg + 60 mg, i.p) to avoid distress to the mice (to make them unconscious and reduce the painful feeling associated with the euthanasia) and then CO2 chamber was used to euthanize the mice. The institutional ethical committee regulated the overall process of euthanasia. Prior to the disposal, the animal death was confirmed by observing the movement, heartbeat, respiration and eye reflex.

RETRACTED

### Randomization, blinding and sample size selection

The animals were assigned to various groups randomly as reported previously [16]. Similarly, to avoid experimental biasness double blindness was maintained during the whole experiment as mentioned [16]. The sample size (*n* = 6–7) was selected according to the previously established protocols [16–19]. At the end of the experiments the mice were euthanized using CO_2_ chamber.

### Acetic acid-induced visceral pain model

Acetic acid-induced writhing test was performed in mice as described previously [20]. The acetic acid-induced pain model simulate the visceral pain model and initiated by the release of inflammatory mediators, which trigger the sensitization of the sensitization of nociceptors [20, 21]. Briefly, acetic acid (0.8% v/v, 10 ml/kg) was injected into peritoneal cavity of the mice. Mice were then placed in large glass cylinder (10 cm diameter) and writhing response was measured i.e. number of writhes occurring between 0 and 30 min after acetic acid injection. Drugs were administered by i.p route 40 min prior to acetic acid induction, control group was treated with vehicle (2% DMSO in 300 μl saline, i.p), positive control was treated with piroxicam (5 mg/kg, i.p) and the treatment group received poncirin (5 mg/kg, 15 mg/kg or 30 mg/kg, i.p).

### Formalin-induced tonic pain model

Paw licking was induced by intraplantar injection of formalin as described previously with some modification [22]. Before the initiation of formalin-induction, the mice were transferred to the formalin testing boxes and observed for 30 min. Following the induction of the formalin-induced nociception, animals were further observed for 30 min and the total time taken was 60 min as reported previously with necessary modification [23]. Mice were observed for first 10 min (early phase) and from 10 to 30 min (late phase) and total time spent in licking the injected paw was calculated for both phases. The mice were administered drugs through i.p. route 40 min prior to formalin induction. Control group was treated with vehicle (2% DMSO in 300 μl saline, i.p) and positive control was treated with piroxicam (5 mg/kg), while treatment group received poncirin (5 mg/kg, 15 mg/kg or 30 mg/kg, i.p).

RETRACTED

### Carrageenan-induced acute inflammatory pain model

The anti-inflammatory potential of the poncirin against the Carrageenan-induced inflammatory model was explored [24]. The animals were randomly divided into various groups as described above. The Carrageenan-induced inflammation was established by injecting 1% carrageenan solution into the right hind paw as reported [24].

### Assessment of mechanical hyperalgesia in carrageenan-induced inflammatory pain

The mechanical hyperalgesia test was performed by using Randall Selitto (Digital Paw Pressure Randall Selitto Meter, IITC Life Science Inc. Wood land Hills, CA) according to the method described previously [24–26]. Animals were pretreated with poncirin (30 mg/kg) or vehicle (2% DMSO in 300 μl saline, i.p) or dexamethasone (5 mg/kg) 1 h before the injection of carrageenan (100 μg/paw). The anti-hyperalgesic response of poncirin was recorded 4 h after the carrageenan injection.

### Assessment of mechanical allodynia in carrageenan-treated mice

In order to evaluate the anti-allodynic effects of poncirin in acute inflammatory pain model was noted 4 h after carrageenan injection (100 μg /paw). One day before the experiment, baseline withdrawal threshold was determined for all animals. On the day of the experiment, animals were treated with poncirin (30 mg/kg) or vehicle (2% DMSO in 300 μl saline, i.p) or dexamethasone (5 mg/kg) 1 h before the injection of carrageenan. Mechanical allodynia was measured in all the treated groups using previously described protocol [27, 28].

### Assessment of thermal hyperalgesia in carrageenan-treated mice

Spontaneous nociception to heat stimuli was measured according to previously described methods [29]. Mice were placed in quiet room 30 min before starting the test and were observed for the signs of the nociception including licking of the hind paws. The response latency was considered as nociceptive behavior with a cut off time of 35 s, in order to avoid any tissue damage.

### Paw edema test in carrageenan-treated mice

Paw edema was measured in carrageenan-induced inflammatory pain model according to the methods previously described [26, 28]. Briefly, paw thickness was measured by using a dial thickness gauge (No. 2046F, Mitutoyo, Kawasaki, Japan) one day before and after carrageenan (100 μg/paw) administration for all the treated groups.

RETRACTED

### CFA-induced chronic inflammatory pain model

For the evaluation of anti-hyperalgesic activity of poncirin in chronic inflammatory pain model, CFA-induced pain model was employed [28, 30]. For the evaluation of the effect of poncirin on acute inflammation and pain, readings were taken at 2, 4 and 6 h post CFA injection. While to investigate the effect of chronic treatment of poncirin on mechanical and thermal sensitivity, mice were treated with poncirin once a day for the period of 6 days. However, the dose of poncirin was skipped at day 5 in order to check any tolerance effects (to see whether the effect of the drug remains persistent or it should be administered daily to achieve the response) as described previously [28].

### Assessment of mechanical hyperalgesia and allodynia induced by CFA

To evaluate mechanical hyperalgesia induced by CFA, mice were treated with poncirin (30 mg/kg), vehicle (2% DMSO in 300 μl saline, i.p) or dexamethasone (5 mg/kg) by intra peritoneal route 40 min before the injection of CFA (20 μl/paw). One day before the experiment, baseline withdrawal threshold was determined for all animals. For the evaluation of acute effects of poncirin on pain profile, readings were taken at 2, 4 and 6 h post CFA injection. Mechanical hyperalgesia was measured by Randall Selitto (Digital Paw Pressure Randall Selitto Meter, IITC Life Science Inc. Wood land Hills, CA), while mechanical allodynia was measured using von Frey hair filament.

### Assessment of thermal hyperalgesia induced by CFA

Hotplate test was carried out in mice model of CFA induced inflammatory pain as described previously [29]. One day before the experiment, baseline withdrawal threshold was determined for all animals. Readings were taken at 2, 4 and 6 h post CFA injection in order to evaluate the effect of poncirin in the acute phase, while readings were taken for 6 consecutive days for the chronic study. The dose of the poncirin was skipped at day 5 to assess the tolerance effect as reported previously [28].

### Assessment of cold allodynia in CFA-treated mice-cold acetone test

Cold acetone test was carried out in mice model of CFA-induced inflammatory pain as described previously [31, 32]. One day before the experiment, baseline withdrawal threshold was determined for all animals. Mice were placed in glass cylinders, and the noxious cold stimulus was applied in form of brief spray of acetone to the ventral surface of the right hind paw. The nociceptive response, which included licking or biting, was measured for 25 s as mentioned earlier [28].

RETRACTED

### Muscle strength and motor activity

The muscle strength of mice was determined by using weights test and Kondziela’s inverted screen tests, in order to assess the effect of poncirin on motor activity of mice [33]. In Kondziela’s screen test, each mouse was placed in the center of wire mesh screen and the screen was inverted, which was held 40–50 cm above the padded surface. Time taken by mice to hold the inverted screen was recorded using a digital stopwatch and score was assigned according to the protocol described elsewhere [33]. Weight test was performed for measuring muscle strength according to the protocol described previously [33].

### Biochemical assays

#### Serum nitrite determination

Griess reagents was used to determine the serum nitric oxide (NO) as reported previously [34, 35]. The blood was centrifuged at 2500 rpm for 10 min following collection of the blood directly from the cardiac puncture and NO was determined as described [34, 35].

#### Extraction of mRNA and q-RT-PCR

At day 6 of the CFA administration the animals were anesthetized with Xylazine + ketamine (16 mg + 60 mg, i.p) to remove the paw tissue. Following removal of paw tissue, the animals were euthanized in the CO2 chamber [36]. Mice paw were used for the extraction of total RNA using Trizol Reagent according to manufacturer instructions (Invitrogen Life Technologies, Carlsbad, CA, USA) as described previously [28]. Briefly, q-RT-PCR analysis for various target genes (TNF-α, IL-1β, IL-6, Nrf2, HO-1, SOD2, VEGF, β-actin) mRNA was performed using Applied Biosystems (AB) detection instruments and software as described previously [28]. The forward and revere primers used are listed in the Table 1.

**Table 1:** the sequences of PCR primers

Genes	Forward primer	Reverse prime
β-actin	TGAAGGTCGGTGTGAACGGATTTGGC	CATGTAGGCCATGAGGTCCACCAC
TNF-α	GTTCTATGGCCCAGACCCTCA	GGCACCACTAGTTGGTTGTCTTTG
IL-1β	TCC AGG ATG AGG ACA TGA GCAC	GAA CGT CAC CCA GCA GGT TA
IL-6	CCA CTT CAC AAG TCG GAG GCT TA	CCA GTT TGG TAG CAT CCA TCA TTT C
VEGF	TTACTGCTGTACCTCCACC	ACAGGACGGCTTGAAGATG
Nrf2	TGG GGA ACC TGT GCT GAG TCA CTG GAG	ACC CCT TGG ACA CGA CTC AGT GAC CTC
HO-1	CACGCATATACCCGCTACCT	CCAGAGTGTTCATTCGAGA
SOD2	GCGGTCGTGTAAACCTCAT	GGTGAGGGTGTCAGAGTGT

#### Renal and liver toxicity

Biochemical tests were performed using serum samples for assessment of RFTs and LFTs (Renal function tests and liver function tests) at day 6 of the CFA administration. Serum Aspartate Aminotransferase (AST), Alanine Aminotransferase (ALT) and creatinine concentration were determined as indicators of liver and kidney functions respectively [37, 38].

RETRACTED

#### Histopathological and X-ray examination of inflamed paws

To observe the effect of daily treatment of poncirin on mice paw tissue, histopathological and radiological analysis of the paw tissues were performed [21]. At day 6 of the CFA administration the animals were anesthetized with Xylazine + ketamine (16 mg/kg + 60 mg/kg, i.p) and were euthanized in the CO2 chamber as mentioned [21]. After removal, each paw was washed using saline and then fixed in 10% formalin solution, dehydrated and embedded in paraffin according to the methods described previously [21]. Paw tissue blocks sections were made of 4 μm thickness, stained with hematoxylin-eosin and observed by microscopy (40×) as per reported protocols [21]. Similarly, the X-ray analysis (Philips 612 machine 40 kW for 0.01 s) was performed as to assess the soft tissue swelling and bone erosion as described previously [21].

### Statistical analysis

All results are expressed as mean ± SEM. The differences between the control and normal groups were tested by one-way analysis of variance (ANOVA) followed by Student’s t-test using SPSS (version 10.0, Chicago, IL). A value of *p* < 0.05 was chosen as the criterion for statistical significance. The graphs were plotted using Sigma plot version 12.0, Chicago, USA.

## Results

### Poncirin inhibits abdominal constriction induced by acetic acid

In the first set of experiments, the anti-nociceptive effect of poncirin was assessed in acetic acid-induced visceral pain (Fig. 1), which has been employed widely for the assessment of anti-inflammatory or analgesic properties of new compounds [39]. Intraperitoneal administration of poncirin 40 min prior to the acetic acid administration considerably (*p* < 0.05) reduced the number of abdominal writhing movements as compared to vehicle-treated group (Fig. 1).

**Fig. 1:** Inhibition of abdominal writhing induced by acetic-acid as described in “Materials and methods”. The total numbers of writhing were evaluated over the period of 30 min. Each column represents the mean ± SEM of 6–7 mice per group. *p < 0.05, **p < 0.01 and ***p < 0.001 denote the significant differences from the negative control group

### Poncirin reduces formalin-induced paw licking in both phases

The anti-nociceptive effect of poncirin was also confirmed by using formalin test, which produces a biphasic response, each phase represents distinct types of pain [40]. The first phase, named as nociceptive phase, is a result of direct stimulation of nociceptors and is mediated centrally, while the second phase is an inflammatory phase, caused by the local release of hyperalgesic and inflammatory mediators [40]. Formalin injection produced biphasic paw licking response with the first phase ranged from 0 to 10 min, while the second phase ranged from 10 to 30 min. Administration of poncirin 40 min prior to formalin-induction significantly reduced the paw licking response dose dependently in both early phase (Fig. 2a) and late phase (Fig. 2b) respectively, however, the dose of 30 mg/kg showed maximum response (*p* < 0.05). The positive control treated with piroxicam (5 mg/kg) also showed the significant anti-nociceptive effect in both phases.

RETRACTED

**Fig. 2:** Inhibition of formalin-induced paw licking and total time spent in paw licking was reduced by poncirin. The total time spent in paw licking was observed for 0–10 min (**a**) and 10–30 min (**b**) after formalin injection. Treatment with piroxicam (5 mg/kg, i.p) was used as a control. Each column represents the mean ± SEM of 6–7 mice per group. *p < 0.05, **p < 0.01 and ***p < 0.001 denote the significant differences from the negative control group

### Poncirin inhibits carrageenan-induced mechanical and thermal hyperalgesia

The compound poncirin was tested in three different doses (5 mg/kg, 15 mg/kg or 30 mg/kg, i.p) in first two set of experiments and 30 mg/kg dose of poncirin produced significant analgesic responses when compared with negative control groups, therefore, poncirin (30 mg/kg) was used in subsequent experiments. Next, the anti-nociceptive effect of poncirin (30 mg/kg, i.p) was assessed in carrageenan-induced acute inflammatory pain model. Poncirin noticeably inhibited (*p* < 0.05) carrageenan-induced mechanical (Fig. 3a) and thermal (Fig. 3b) hyperalgesia at given dose after 4 h of carrageenan injection. In vehicle-treated group marked increase in pain sensitivity was observed in mechanical (Fig. 3a) and thermal hyperalgesia (Fig. 3b). Whereas, the dexamethasone used as positive control also inhibited mechanical and thermal hyperalgesia (Fig. 3).

**Fig. 3:** Anti-hyperalgesic activities of poncirin in acute inflammatory pain model induced by carrageenan (**a**) inhibition of mechanical hyperalgesia, (**b**) inhibition of thermal hyperalgesia, (**c**) inhibition of mechanical allodynia and (**d**) reduction in paw thickness. Each column represents the mean ± SEM of 6–7 mice per group. *p < 0.05, **p < 0.01 and ***p < 0.001 denote the significant differences from the negative control group

### Poncirin inhibits carrageenan-induced mechanical allodynia and paw edema

The poncirin treatment significantly inhibited carrageenan-induced mechanical allodynia, while the maximum increase in pain threshold (*p* < 0.05) was noticed with escalated dose i.e. 30 mg/kg (Fig. 3c). The positive control (dexamethasone 5 mg/kg, i.p) also exhibited significant reduction in allodynic responses compared, however, the negative control group showed decreased in pain threshold and hypersensitivity to the allodynic stimulus. Similarly, the poncirin administration markedly reversed the carrageenan-induced paw swelling compared to the negative control group (treated with carrageenan only) (Fig. 3d). Furthermore, the positive control group also significantly inhibited the carrageenan-induced paw edema in mice (Fig. 3d).

RETRACTED

### Poncirin inhibits CFA-induced mechanical hyperalgesia and allodynia

Next, the modulatory effect of poncirin was evaluated in mechanical hyperalgesia and allodynia. In order to investigate the effects of poncirin in CFA-induced mechanical hyperalgesia, animals were treated with poncirin (30 mg/kg, i.p) 40 min prior to CFA injection. Poncirin significantly increased pain thresholds in both mechanical hyperalgesia test and allodynia at 2, 4 and 6 h after CFA injection, showing the promising activity of poncirin in acute case. Dexamethasone also significantly increased the pain threshold as compared to negative control (Fig. 4).

**Fig. 4:** Anti-hyperalgesic activities of poncirin in chronic inflammatory pain model induced by CFA (**a**) inhibition of acute mechanical hyperalgesia, (**b**) inhibition of acute mechanical allodynia, (**c**) inhibition of chronic mechanical hyperalgesia and (**d**) inhibition of chronic mechanical allodynia. Each data point represents the mean ± SEM of 6–7 mice per group. *p < 0.05, **p < 0.01 and ***p < 0.001 denote the significant differences from the negative control group

In order to investigate the chronic anti-inflammatory and analgesic effects of poncirin on mechanical hyperalgesia and allodynia, animals were treated daily for 6 days skipping day 5 after CFA injection. Poncirin (30 mg/kg, i.p) daily treatment significantly increased pain thresholds throughout treatment period compared with negative control (Fig. 4c and d) indicating the effectiveness of poncirin in chronic inflammatory pain model. The dose of the poncirin was skipped at day 5 to observe the tolerance effect (whether the anti-inflammatory effect of the poncirin remains persistent while skipping the dose or it should be administered daily to produce its effect) as described previously [28]. However, the poncirin treatment did not exhibited any tolerance effect and the mechanical hyperalgesia and allodynia was reestablished when the dose was skipped at day 5 (Fig. 4c & d).

### Inhibition of thermal hyperalgesia and cold allodynia by poncirin in CFA-induced pain model

In order to investigate the effects of poncirin in CFA-induced thermal hyperalgesia and cold allodynia, animals were treated with poncirin (30 mg/kg, i.p) 40 min prior to CFA injection. Poncirin significantly inhibited acute thermal hyperalgesia (Fig. 5a) at 2, 4 and 6 h after CFA injection, showing the promising activity of poncirin. Dexamethasone treated group also significantly increased the pain threshold as compared to negative control. For long-term effects of poncirin on thermal hyperalgesia, animals were treated daily for 6 days after CFA injection, skipping day 5 for evaluation of tolerance effect (whether the anti-inflammatory effect of the poncirin remains persistent while skipping the dose or it should be administered daily to produce its effect) of the drug on thermal hyperalgesia as reported previously [28]. Poncirin (30 mg/kg, i.p) daily treatment significantly increased pain thresholds (Fig. 5b) indicating the effectiveness of poncirin in chronic inflammatory pain model.

RETRACTED

**Fig. 5:** Anti-nociceptive activities of poncirin in thermal hyperalgesia and cold allodynia induced by CFA (**a**) inhibition of acute thermal hyperalgesia, (**b**) inhibition of chronic thermal hyperalgesia and (**c**) inhibition of cold allodynia. Each data point represents the mean ± SEM of 6–7 mice per group. *p < 0.05, **p < 0.01 and ***p < 0.001 denote the significant differences from the negative control group

Similarly, poncirin significantly inhibited acute cold allodynia (Fig. 5c) at 4 and 6 h after CFA injection. For long-term effects of poncirin on cold allodynia, animals were treated daily for 6 days after CFA injection. Poncirin (30 mg/kg, i.p) daily treatment significantly increased pain thresholds on day 4 and 6 compared with negative control, indicating the effectiveness of poncirin in chronic inflammatory pain model (Fig. 5c).

### Poncirin inhibited CFA-induced paw edema

Poncirin inhibited paw edema induced by CFA in both acute and chronic inflammation models. Administration of poncirin significantly reduced the paw thickness at 2, 4 and 6 h after CFA-induced acute edema (Fig. 6a). For the evaluation of long-term effects of poncirin in CFA-induced paw edema, poncirin (30 mg/kg) treatment for 6 days showed significant inhibition of paw edema compared to CFA treated group (Fig. 6b). Similarly, the positive control (dexamethasone 5 mg/kg) also significantly attenuated the acute paw edema 2, 4 and 6 h after CFA administration, while the daily administration of dexamethasone (5 mg/kg) for 6 days also markedly attenuated the CFA-induced paw edema compared to the negative control (Fig. 6b).

**Fig. 6:** Anti-inflammatory activities of poncirin in paw induced by CFA (**a**) inhibition of acute paw edema and (**b**) inhibition of chronic paw edema. Each data point represents the mean ± SEM of 6–7 mice per group. *p < 0.05, **p < 0.01 and ***p < 0.001 denote the significant differences from the negative control group

RETRACTED

### Poncirin doesn’t have any effect on the motor activity of mice

Poncirin chronic administration does not effected the motor function of the mice, which was evaluated by Weights test and Kondziela’s screen tests utilized as a screening tool in preliminary drug research for evaluation of motor function (Fig. 7a and b) [33, 41]. Motor function was altered in the CFA-treated group while both poncirin and dexamethasone did not alter the muscle strength both after acute and long-term administration of drugs.

**Fig. 7:** (**a**) Effect of poncirin treatment on muscle strength and motor coordination of animals was measured by using inverted tray method at 0 h, 6 h and day 6 as described in materials and method section. (**b**) Effect of poncirin treatment on muscle coordination of animals was measured by using weight test at 0 h, 6 h, and day 6. Each column represents the means ± SEM of 6–7 mice per group. *p < 0.05, **p < 0.01 and ***p < 0.001 denote the significant differences from the negative control group

### Body weight assessment

Each group of mice were weighted before the disease induction with CFA. Similarly, the weight of mice were also recorded at day 6 of the CFA administration at the end of the experiment as shown (Additional file 1).

### Poncirin reduced the production of NO in plasma after CFA induction

The inhibitory effect of poncirin on NO production in plasma was analyzed on day 6 of the CFA administration using Griess reagent method as described previously [28]. The CFA administration markedly increased the production of NO in mice plasma at day 6 of the administration. The poncirin (30 mg/kg) treatment significantly attenuated the NO (almost 80%) production compared to the negative control (only CFA treated group) (Fig. 8). Similarly, the dexamethasone-treated group also showed obvious decrease in NO production (approximately 83% decrease was noted in NO production) (Fig. 8).

**Fig. 8:** Effect of treatment with poncirin on nitrite (NO) production determination in blood plasma. Each column represents the means ± SEM of 6–7 mice per group. *p < 0.05, **p < 0.01 and ***p < 0.001 denote the significant differences from the negative control group

### Poncirin inhibits CFA-induced pro-inflammatory cytokines production

To examine the effect of poncirin (30 mg/kg) on the production of pro-inflammatory cytokines in CFA-treated paw, qRT- PCR was performed. qRT-PCR results showed increased expressions of TNF-α, IL-1β, IL-6 and VEGF mRNA in CFA-induced mice paw tissue (Fig. 9a, b, c and d). Whereas, poncirin treatment strikingly inhibited the mRNA expression levels of pro-algesic and inflammatory cytokines such as TNF-α, IL-1β, IL-6 and VEGF (Fig. 9).

RETRACTED

**Fig. 9:** (**a**) Effect of treatment with poncirin on mRNA expression levels of TNF-α, (**b**) IL-6, (**c**) IL-1β and (**d**) VEGF in mice paw tissue. The mice were treated with poncirin (30 mg/kg, i.p), dexamethasone (5 mg/kg, i.p) or vehicle control as described in “Materials and methods”. Each column represents the mean ± SEM of 6–7 mice per group. *p < 0.05, ** *p* < 0.01 and ***p < 0.001 denote the significant differences from the negative control group

### Poncirin increased the expression levels of Nrf2, HO-1, and SOD2 in CFA-induced inflammatory pain model

qRT-PCR was also used to investigate the effect of poncirin treatment on expression levels of the phase II antioxidant enzymes (HO-1 and SOD2). Nrf2 activates antioxidant response element (ARE) that in turns is responsible for the expression of phase II antioxidant enzymes [42]. The mRNA expression levels of SOD2 (approximately 79% increase was noticed) and HO-1 (more than 5 times) was increased in poncirin treated group as compared to CFA treated group (Fig. 10b and c). Poncirin treatment up-regulated Nrf2 (100% increase) expression level considerably (Fig. 10a).

**Fig. 10:** (**a**) Effect of treatment with poncirin on protein expression of Nrf2, (**b**) HO-1 and (**c**) SOD2 in mice paw tissue. Each column represents the means ± SEM of 6–7 mice per group. *p < 0.05, **p < 0.01 and ***p < 0.001 denote the significant differences from the negative control group

### Poncirin doesn’t cause hepatic or renal damage

Mice were treated daily with poncirin (30 mg/kg, i.p) or dexamethasone (5 mg/kg, i.p) or vehicle for 6 days after induction of inflammatory pain. The treatment with poncirin and dexamethasone did not alter the hepatic and renal functions (Table 2), thus signifies that poncirin administration did not produce any toxicity against these vital organs.

**Table 2:** Effect of poncirin on liver and kidney function

Sample	Creatinine (mg/dL)	GPT/ALT (UI/L)	GOT/AST (UI/L)
Normal	0.4 ± 0.28	94 ± 1.41	141 ± 2.82
Dex 5 mg/kg	0.4 ± 0.22	94 ± 1.56	142 ± 1.25
Poncirin 30 mg/kg	0.4 ± 0.14	95 ± 2.12	144 ± 2.12

### Poncirin inhibited infiltration of inflammatory cells and soft tissue swelling after CFA induction

Histopathological analysis of tibiotarsal joints of right hind paw showed a significant infiltration of immune cells and synovial hyperplasia in CFA treated group, while poncirin treated group showed a reduction of immune cells infiltration and synovial hyperplasia (Fig. 11b). The radiographic examination of the soft tissue showed marked reduction in soft tissue swelling of the right hind paw in those animals who were treated with the poncirin, however, the animals challenged with CFA only showed noticeable soft tissue swelling and bony erosion (Fig. 11a).

RETRACTED

**Fig. 11:** Clinical appearance of right hind paws. (**a**) Radiographic evidence of right hind paw from (1) Vehicle control, (2) negative control group, (3) positive control group and (4) poncirin treated group. Tissue swelling can be observed in the tibiotarsal region of CFA treated mice as compared to poncirin treated mice. (**b**) Histopathological analysis of tibiotarsal joint from (1) vehicle control, (2) negative control group, (3) positive control treated group and (4) poncirin treated group. Paw tissues were sectioned at 4 μm thickness, stained by hematoxylin-eosin and observed with the microscope (40×). Note marked immune cell infiltration, synovial hyperplasia, in the vehicle-treated group as compared to poncirin treated group

## Discussion

Inflammatory pain is a common chief complaint associated with many disease conditions including irritable bowel syndrome, rheumatoid arthritis and osteoarthritis [2]. The inflammation mediated pain trigger the induction of pro-inflammatory cytokines and activates several signaling pathways such as NF-κB, MAPKs etc. Currently, several therapeutic approaches are employed to treat the inflammatory pain such as NSAIDs and opioids [43]. The chronic use of NSAIDs such as aspirin can cause the GIT ulceration, while the prolonged use of opioids is related with the development of tolerance, dependence and respiratory depression [44–47]. All these challenges necessitate the development and discovery new molecules, which are safe, effective and associated with less side effects profile. Since decades, medicinal plants have been used for therapeutic purposes, as they are effective and safe and offer a good source of new chemical entity [44–47]. Poncirin is flavanone derivative obtained from dried immature fruits of *Poncirus trifoliata*, which was used to treat inflammation and asthma in ancient times [44–47]. Recent studies on poncirin have also confirmed its anticancer and anti-inflammatory activity [14]. In the current study, it was demonstrated that systemic administration of poncirin in various inflammatory pain models successfully alleviated pain associated with inflammation. The anti-hyperalgesic effects of poncirin in inflammatory pain can be attributed to suppression of pro-inflammatory cytokines including TNF-α, IL-1β and IL-6, enhancing the expression of antioxidant genes and enzymes (Nrf2, HO-1 and SOD2) respectively. Therefore, the present study highlights the analgesic potential of poncirin together with its safety since the systemic administration of poncirin did not present any renal, hepatic or motor side effects.

RETRACTED

Acetic acid-induced abdominal writhing is a simple method for novel drugs screening in visceral pain [20]. Acetic acid administration causes the activation of peritoneal macrophages and mast cells which leads to local release cytokines such as TNF-α and IL-1β and other mediators like eicosanoids and sympathomimetic amines [38]. Since poncirin administration inhibited acetic acid-induced writhing markedly, it is likely that the anti-nociceptive activity of poncirin might be contributed due to its inhibitory activity cytokines production. Similarly, the anti-nociceptive activity of poncirin was also observed in formalin-induced tonic pain model. The injection of formalin causes an intense and immediate increase in impulses transmission from C afferent fibers and produce a diverse quantifiable behavior as paw licking by the animal that indicates the intensity of pain [48]. This test can also be used to determine the effect of new compounds on central and peripheral nociceptive pathways as formalin injection causes biphasic reaction consisting of early neurogenic phase and late inflammatory phase [49]. The early neurogenic phase of formalin injection last from 0 to 10 min and is caused by the release of neurotransmitters such bradykinin and serotonin as well as molecules released from residents cells causing the activation of transient receptor potential ankyrin 1 (TRPA1) on the surface of nociceptive fibers [50]. The late inflammatory phase of formalin test lasts from 10 to 30 min and occurs because of release of inflammatory cytokines including TNF-α, IL-1β, IL-6 and prostaglandins after administration of inflammatory stimuli like formalin [51]. Poncirin inhibited both paw licking and total time spent in paw licking in both phases of formalin injection. Interestingly, poncirin administration reduced the total spent in paw licking in the first phase as compared the positive control, showing its effect on the central pain pathways. The analgesic potential of poncirin was also demonstrated in carrageenan- and CFA-induced acute and chronic inflammatory pain models. Carrageenan and CFA are algogenic substances and cause the local release of mediators, such as prostanoids and cytokines, involved in the inflammatory signs such as vasodilation, edema, and hyperalgesia [52, 53]. Importantly, the systemic administration of poncirin reduced both hyperalgesia and allodynia in both carrageenan and CFA model with comparable results to dexamethasone, which is a standard anti-inflammatory drug, showing the anti-nociceptive potential of poncirin. Carrageenan- and CFA-induced inflammatory pain are well-accepted models of acute and chronic pain respectively. The peripheral injection of algogenic substances like carrageenan and CFA causes the release of numerous nociceptive and inflammatory mediators, resulting in the alteration of synaptic activity by increasing the primary sensory fibers discharge and causing central pain sensitization by modifying neuroimmune cells [54]. In present study, systemic administration of flavanone glycoside poncirin remarkably inhibited the mechanical, thermal hyperalgesia and mechanical and cold allodynia induced by carrageenan and CFA in both acute and chronic inflammation models in mice. Poncirin increased the pain threshold after 2 h of treatment and its effects persisted until 6 h in the acute model and until day 5 in the chronic model. The paw edema induced by carrageenan and CFA was also significantly reduced by poncirin. Because TNF-α, IL-1β and IL-6, play a key role in inflammatory hyperalgesia, it may be suggested that the anti-nociceptive effects of poncirin are due to its ability to inhibit the release of inflammatory cytokines [44].

RETRACTED

NO is a well-established mediator of inflammation and its production is related to the degree of inflammation [55]. The expression of NO is under the influence of iNOS gene, however, its production is also regulated by the TNF-α, thus maintain the hyperalgesic state after the inflammation and pain. The poncirin treatment significantly reduced the levels of NO compared to the CFA-induced group.

Inflammation is closely related to sensation of pain [5]. Following the local injection of CFA there is a release of various inflammatory mediators including TNF-α, IL-1β and IL-6. NO also contributes to the hyperalgesic state by indirectly sensitizing the nociceptors through the production of prostanoids such as PGE2. In addition, these cytokines increase the synaptic transmission by directly activating nociceptors [4]. In the present study, poncirin also significantly reduced the expression of TNF-α, IL-1β and IL-6 in CFA induced inflammatory pain, suggesting that suppression of these pro-inflammatory cytokines contributes to the anti-nociceptive activity of poncirin. Vascular endothelial growth factor (VEGF) induces vascular leakage by enhancing vascular permeability, thus playing an important role in inflammation [56]. The expression of inflammatory cytokines is, also induced by VEGF indicating the role of VEGF in the production of these hyperalgesic cytokines [56]. The poncirin treatment significantly reduced the mRNA expression level of the VEGF compared to the negative control group, thus, indicating the potent anti-inflammatory role of the poncirin.

RETRACTED

Nrf2 is transcription factor responsible for the induction antioxidant enzymes including glutathione peroxidase (GPx), Glutathione S transferase (GST) and HO-1 [42]. Nrf2 have multiple protective actions including antioxidant activity by induction of antioxidant enzymes, anti-inflammatory role in many diseases as well as protective action in wound healing [57, 58]. The protective anti-inflammatory role of Nrf2 is attributed to inhibition of expression of pro-inflammatory cytokines, iNOS and COX-2 in early events of inflammation. HO-1 is one of the major anti-inflammatory and cytoprotective enzymes, expression of which is controlled by Nrf2 [59]. The HO-1 expression is induced by many inflammatory stimuli and increased inflammatory state was observed in mice deficient with HO-1 emphasizing on the important role of HO-1 in inflammation resolution and hence decreasing hyperalgesic state [60]. In the current study, systemic administration of poncirin has shown to significantly increased the expression of Nrf2 and induction of HO-1, highlighting its importance in reducing the inflammatory pain through Nrf2 mediated pathway. Poncirin treatment also up-regulated the expression of SOD2 (superoxide dismutase 2) following CFA-induced inflammatory pain in mice. SOD2 is antioxidant enzyme belonging to SOD family and plays important role in body defense as antioxidant enzyme by modulating the production of inflammatory cytokines [61]. SOD2 high levels in the body inhibit the phospholipase-2 (PLA2) overexpression and consequently inhibits the downstream PGE2 production via NF-κB-dependent pathways [62], thus, reduces the pain by reducing the inflammation.

To assess the toxic effect of poncirin on liver and kidney, liver and kidney functions test were performed using blood plasma. The poncirin treatment exhibits no toxic effect on the liver and kidney. Similarly, to observe any possible toxic effect on the animals, muscle strength and coordination was assessed. The poncirin treatment was not associated with any toxic effect on the muscle strength and coordination.

## Conclusion

Poncirin significantly reduced abdominal writhing in acetic acid-induced visceral pain and also showed remarkable results in both phases of formalin test. In addition, poncirin administration also significantly produced anti-allodynic and anti-hyperalgesic effects in carrageenan- and CFA-induced models. Importantly, chronic treatment with poncirin in CFA model did not produce any side effects. Poncirin also reduced the NO content and pro-inflammatory cytokines expression including TNF-α, IL-1β and IL-6 in paw tissue. The mRNA expression of VEGF was also inhibited by poncirin, which correlates to reduction in paw edema and increased pain thresholds in CFA induced inflammatory pain models. Poncirin also significantly increased the antioxidant enzymes (HO-1 and SOD2) and transcription factor (Nrf2), suggesting that protective role of poncirin as well as multiple targets by which poncirin modulates pain. Collectively, our data demonstrate the analgesic potential of poncirin in acute and chronic inflammatory pain conditions that still need an effective and safe therapeutic option.

RETRACTED

## Additional file

Additional file 1: **Figure S1.** Body weight assessment. The weight of animals at day 1 and day 7. (DOCX 59 kb)

## Data Availability

The data used in the current study can be accessed by requesting the corresponding author.

## Abbreviations

CFA: Complete Freund’s adjuvant
COX-2: Cyclooxygenase-2
CREB: cAMP response element-binding protein
Dex: Dexamethasone
HO-1: Heme oxygenase
i.p.: intraperitoneal
i.pl: intraplantar
IκB: Inhibitory kappa B
MAPKs: Mitogen activated protein kinase
NF-κB: Nuclear factor kappa B
NO: Nitric oxide
Nrf2: Nuclear factor (erythroid-derived 2)-like 2
SOD2: Superoxide dismutase
